This article has been retracted.

# Role of Nanoparticles in Environmental Remediation: An Insight into Heavy Metal Pollution from Dentistry

**DOI:** 10.1155/2022/1946724

**Published:** 2022-03-17

**Authors:** Lakshmi Thangavelu, Geetha Royapuram Veeraragavan, Sreekanth Kumar Mallineni, Ezhilarasan Devaraj, Royapuram Parthasarathy Parameswari, Nazmul Huda Syed, Kamal Dua, Dinesh Kumar Chellappan, Sri Renukadevi Balusamy, Ujjal K. Bhawal

**Affiliations:** ^1^Department of Pharmacology, Mandy Dental College, University of Dhaka, Dhaka, Bangladesh; ^2^Center for Transdisciplinary Research, Department of Pharmacology, Saveetha Dental College, Saveetha Institute of Medical and Technical Science, Saveetha University, Chennai, India; ^3^Department of Microbiology, Saveetha Dental College, Saveetha Institute of Medical and Technical Sciences (SIMATS), Saveetha University, Chennai, Tamil Nadu 600 077, India; ^4^Department of Preventive Dental Sciences, College of Dentistry, Majmaah University, Almajmaah 11952, Saudi Arabia; ^5^Department of Ophthalmology and Visual Science, School of Medical Sciences, Health Campus, Universiti Sains Malaysia, Kubang Kerian, George Town 16150, Kelantan, Malaysia; ^6^Discipline of Pharmacy, Graduate School of Health, University of Technology Sydney, Sydney, NSW 2007, Australia; ^7^Department of Life Sciences, School of Pharmacy, International Medical University, Bukit Jalil, Kuala Lumpur 57000, Malaysia; ^8^Department of Food Science and Biotechnology, Sejong University, Gwangjin-gu, Seoul 05006, Republic of Korea; ^9^Department of Biochemistry and Molecular Biology, Nihon University School of Dentistry at Matsudo, Chiba 271-8587, Japan

## Abstract

Environmental damage is without a doubt one of the most serious issues confronting society today. As dental professionals, we must recognize that some of the procedures and techniques we have been using may pose environmental risks. The usage and discharge of heavy metals from dental set-ups pollute the environment and pose a serious threat to the ecosystem. Due to the exclusive properties of nanosized particles, nanotechnology is a booming field that is being extensively studied for the remediation of pollutants. Given that the nanoparticles have a high surface area to volume ratio and significantly greater reactivity, they have been greatly considered for environmental remediation. This review aims at identifying the heavy metal sources and their environmental impact in dentistry and provides insights into the usage of nanoparticles in environmental remediation. Although the literature on various functions of inorganic nanoparticles in environmental remediation was reviewed, the research is still confined to laboratory set-ups and there is a need for more studies on the usage of nanoparticles in environmental remediation.

## 1. Introduction

Environmental pollution is one of the major concerns for the international community currently. The rapid industrial and economic development has resulted in increased energy consumption, as well as the release of toxic gas emissions and hazardous waste into the environment [1]. The environment is contaminated by different pollutants such as organometallic compounds, inorganic metal ions, organic contaminants, and nanoparticles, including heavy metals [2]. The name “heavy metal” is because of their high density and atomic weight. Recently, they are described as metallic chemical elements and metalloids that cause a serious hazard to human well-being and the environment even at low concentrations [3, 4]. To accomplish the professional goals in dentistry, dentists utilize a range of materials and tools. Unfortunately, certain constituents, such as biomedical waste and the use of heavy metals, pose a possible threat to the ecosystem. One such material, dental amalgam containing mercury, silver, and various other heavy metals, has been extensively used as a metallic restorative substance in dentistry. Given its high content of mercury, the safety of its usage is controversial [5, 6]. Dental waste is collected along with household and municipal waste and is released into the environment to pollute soil, water, and air [7]. Therefore, dental practitioners have recently been more concerned about the environmental pollution caused by dentistry and various methods employed to tackle it.

Nanomaterials are small materials with at least one dimension measuring under 100 nm [8]. Due to their small size and large reactive surfaces, they are very good catalysts and adsorbents [9, 10]. In parallel to the conventional technologies, the swift growth of nanotechnology has developed a great concern in the use of nanomaterials in environmental remediation. These distinctive characteristics along with cost-effectivity are used effectively to remove and degrade contaminants from the environment [11]. In this review, we aim to introduce and describe the heavy metal pollution from dentistry and nanoparticles with deeper insights into their types and their roles in environmental remediation.

## 2. Heavy Metal Pollution from Dentistry and Their Environmental Effects

To meet increasing awareness and responsibilities towards the environment, dental professionals should be mindful of environmental impact from clinical practice. Although dentists individually produce just a small amount of hazardous waste, the trash accumulated by the whole profession might have a serious effect on the environment [12]. One of the major concerns in recent years is the effect of heavy metal contamination of water bodies, especially through the release of dental amalgam. Amalgam contains silver, copper, tin, and, mostly, mercury that can enter the ecosystem [13, 14]. Amalgam scarp management might cause soil pollution, whereas the effluents released from dental clinics pollute the water.  Figure 1 shows the heavy metal sources in dentistry causing pollution.

*Mercury* accounts for up to 50% of the weight of amalgam restorations [15]. Mercury bioaccumulates and is known to cause harmful effects in humans and nature [16]. Dental amalgam mercury can harm the environment in several ways such as wastewater from dental offices, human waste, and mercury vapour. Benaissa et al. well documented the concentrations of heavy metals from dentistry in wastewater and reported elevated levels of heavy metals in the wastewater from dental clinics exceeding the permitted threshold limits in the region. The concentration of mercury was highest among all the samples of the study. Furthermore, the mercury in amalgam waste was also reported to be hazardous to the environment [17]. Once in the environment, bacteria can convert it into more toxic organic form methylmercury [18]. This organic form of mercury can enter the food web and cause adverse effects among the living organisms [19]. Some of the oral manifestations include osteitis, gingivitis, ptyalism, and ulcers of the oral cavity [20].

*Silver* is an additional heavy metal that can flow into the environment through inappropriate discarding of dental waste. It can be present in various kinds of wastes in a dental facility. Along with amalgam, it can also be found in X-ray fixers and films [21]. Dental fixer solutions use silver thiosulphate complexes that are reported to be 17,500 times less lethal than unbound silver ions [22]. Although a minimum quantity of silver waste is generated from dental clinics, most wastewater agencies mandate pretreatment and levy restrictions on the quantity of silver in wastewater [23].

*Lead* is another common waste from dental practices that must be properly disposed of. Lead shields that are present in film packets are the by-product of conventional radiography. It can also be found in aprons and collars that are used to reduce radiation exposure during X-ray procedures. Although the amount is relatively small, the total waste produced can be significant [24]. Even in the little amounts, it is toxic to the environment and causes adverse health effects to both children and adults. Dental practitioners can easily reduce the environmental contamination of lead by recycling the lead shields from film packets. In addition, several other toxic heavy metals such as zirconium, cobalt, and chromium are extensively used in dentistry posing a serious threat to the environment [25].

Life cycle assessment (LCA) can be used as a means to measure the environmental impact associated with the stages of the life cycle (mining, purification, and refining) of a product such as heavy metals. Data from life cycle inventory (LCI) databases provide substantial information on the life cycle wide energy use and larger environmental impacts of metals [26]. It was reported that, if compared on a per kilogram basis, platinum group metals and gold present the highest burden on the environment, whereas iron, manganese, and titanium were found to have lower environmental impact. Comparing their global annual production in the year 2008, iron and aluminium had highest impacts. The environmental impact of the majority of the elements was dominated by the purification and refining stages [27].

## 3. Nanoparticles in Dentistry

Over the years, progress in dentistry has made dental procedures reliable, safe, fast, and painless. Technologies such as nanotechnology are said to have a great impact on recovery times and treatment methodologies. They possess improved properties, usually because of their quantum effects and rise in surface area [28]. Nanotechnology and nanomaterials provide significant scope in dentistry to enhance dental care, treatment, and the prevention of oral diseases. Various fields of dentistry where nanoparticles have been extensively studied are shown in Figure 2. In general, they are being used as tooth sealers, fillers, and restorative composite materials to improve oral health. Furthermore, nanoparticles-based drug release systems are employed in the targeted therapy of dental diseases. The various applications of nanomaterials across different domains of dentistry are described in the below sections. Some of the current applications of nanoparticles across various branches of dentistry are listed in Table 1.

### 3.1. Periodontal Treatment

Diseases that involve gingiva, alveolar bone, and the surrounding connective tissue are referred to as periodontal diseases [47]. Nanomaterials can be used to deliver the encapsulated drug molecules to the area of interest affected by periodontal disease. Thus, reducing the dosage-related side effects by timely release of drugs to the localized areas affected [32]. Nanomaterials that are experimented for regulated drug release comprise hollow spheres, nanotubes, nanocomposite, and core-shell structure [28]. Chitosan is a naturally occurring polymer that is considered suitable for the treatment of periodontitis due to its antimicrobial properties and the ability to deliver antiseptic drugs to the affected site [48]. Periodontal inflammation treated with triclosan-loaded nanoparticles has been demonstrated to be successful in treating periodontal inflammation [29]. An in vivo report in mice showed that nanostructured doxycycline gel protected the periodontal exterior following empirically induced periodontal disease [31]. Moreover, nanorobots are configured to be area-specific and could be used to destroy bacteria in plaque [32].

### 3.2. Endodontic Treatment

Endodontics involves the treatment of tooth pulp, a loose connective tissue that forms and supports dentine in the centre of the tooth [49]. Nanotechnology is being applied to the field of endodontics as well. Microorganisms tend to resist the root canal treatment and may cause secondary infections throughout or after the filling [49]. Lately, Markan et al. have stated nanoparticle-based disinfection with chitosan, zinc oxide, and silver for the effective removal of microorganisms [33]. Under UV illumination, zinc oxide nanoparticles produce reactive oxygen species (ROS) such as hydroxyl radicals, hydrogen peroxide (H_2_O_2_), and superoxide (O^2^). Hydrogen peroxide molecules have the ability to pass across the cell wall and produce oxidative injury to cellular arrangements [50].

A silicon-based sealer containing silver nanoparticles and a bioceramic-based sealer containing calcium silicate, zirconia, and calcium phosphate are recently been used to enhance the handling, biocompatibility, and physical properties [51, 52]. In a regenerative endodontic approach, nanoscale assemblies of polyglutamic acid (PGA) and poly-l-lysine (DGL) have been used along with an anti-inflammatory hormone to reduce dental pulp inflammation and promote regeneration of pulp fibroblasts [34, 35].

### 3.3. Orthodontic Treatment

Orthodontics includes corrective treatment of teeth that are irregularly positioned by mechanical means to set up satisfactory facial contours [53]. The usage of braces results in white spot lesion development [54]. Nanomaterials such as titanium oxide and silver have been combined with the orthodontic brackets for their antibacterial effects [36]. Furthermore, in order to reduce the friction and efficient movement of tooth, inorganic fullerene-like nanoparticles have been coated as dry lubricants on orthodontic wires [37]. Moreover, alumina nanomaterials have been added to increase the mechanical strength of plastic polymer braces [38].

### 3.4. Prosthodontic Treatment

Prosthodontics involves the restoration and replacement of teeth and related soft and hard tissues using dentures, implants, and maxillofacial prosthetics [55]. Poly(methyl methacrylate) (PMMA) is most commonly used denture material [56]. However, there are issues related to its use, such as surface porosity, mucosa irritation, and polymer wearing-off [57]. The application of nanoparticles, for instance, iron or titanium dioxide, has been demonstrated to decrease the porosity of PMMA, thus reducing the plaque accumulation [40]. In order to enhance mechanical properties, for instance, flexural strength, hardness, and low polymerization shrinkage, nanomaterials such as zirconium dioxide, alumina, and carbon nanotubes have been used [39, 58, 59].

### 3.5. Restorative Dentistry

Nanoparticles have recently been used in remineralization, regeneration, and preventive dentistry. The crystal size of nanoparticles is more similar to natural teeth. Nanoparticles such as hydroxyapatite (HA) and anhydrous calcium phosphate (ACP) were reported to have related morphology and substance composition to that of tooth enamel. Therefore, due to their increased surface area for binding, HA nanoparticles are capable to serve as fillers to fix small dents on enamel [41, 42]. Recently, more efforts have been emphasized on developing a strong and durable dental nanocomposite. Hybridization of ACP filler using tetraethoxysilane (TEOS) was reported to enhance the biaxial flexural power of composites with ACP fillers [60]. Furthermore, bioactive glass nanoparticles are reported to have outstanding regenerative properties in dentin mineralization and treating dentine hypersensitivity [43, 61]. In addition, hybrid nanomaterials such as silver fluoride and sodium fluoride in combination with chitosan have been developed for the continuous delivery of the antimicrobial drugs and improved similarity towards enamel [44, 45].

Nanomaterials are also employed in dental pulp cell regeneration. Nanofibers-based scaffolds of type 1 collagen or fibronectin are used for pulp regeneration. The nanofibers act as a mesh for the supported growth of pulpal cells [46, 62]. An injectable collagen scaffold with dental stem cells leads to the building of pulp-like tissue [63].

In addition to the applications of nanomaterials, there remain many research gaps concerning their usage in dentistry. Ensuring key physical, mechanical, and chemical properties of the dental implant and its surface modification is crucial towards studying its therapeutic efficacy. Though the concept of drug delivery has gained attention, it has largely remained constrained to in vitro studies for a short-term release of drugs lasting only a few weeks. It is observed that several cells and proteins tend to cover and block the surface of a drug-releasing implant when placed, thereby impacting the drug delivery. In addition, it is important to determine and control the usage of metal ions and nanomaterials as augmenting agents in order to reduce cytotoxicity.

## 4. Types of Nanoparticles

Nanomaterials are described as substances with at least one dimension ranging from 1 to 100 nm [64]. There are three different categories of nanomaterials like nanoparticles, nanoclay, and nanoemulsions (Figure 3). Nanoparticles are the commonly studied nanomaterials, which are further allocated into organic nanoparticles and inorganic nanoparticles [65].

### 4.1. Organic Nanoparticles

Natural or synthetic organic molecules serve as templates for organic nanoparticles [66]. They have been extensively used in the clinical setting. They were created primarily for drug delivery to avoid the chance of long-lasting toxicity caused by nondegradable polymers. The necessity for organic nanoparticles such as dendrimers, liposomes, polymer micelles, and carbon nanomaterials was understood long since [67, 68]. The key trait of organic nanoparticles is that they provide comparatively simple routes for drug encapsulation [66].

Chitosan is a naturally occurring biocompatible and biodegradable polymer derived from chitin. It has been used as a potential drug delivery vehicle, presenting many advantages. Chitosan can be modified using simple preparation methods to prepare chitosan nanoparticles that can be used in the delivery of numerous drugs for the treatment of several diseases. Chitosan nanoparticles have many advantages, including low toxicity and flexible administration routes [69].

### 4.2. Inorganic Nanoparticles

Inorganic nanoparticles are said to be harmless, biocompatible, and very steady compared with organic nanoparticles and are reported to have adjustable surface and size modification strategies in drug delivery systems [65, 70]. They contain a metal oxide or a metallic particle inside an inorganic core and an outer organic shell. Inorganic nanoparticles are widely used for bioimaging; drug release; therapeutics, for instance, cancer treatment; and dental composites [71–73].

*Gold nanoparticles (GNPs)* are extensively consumed for biomedical applications because of their unique and multisurface functionalities [74]. Unlike gold particles, the colour of GNPs differs from red to purple depending on different masses ranging between 1 nm and 100 nm and distinct forms [65, 75]. The various shapes of GNPs include nanospheres, nanoshells, nanorods, and nanocages. The gold core of GNPs defines the basic characteristics, whereas the surrounding coating can be altered for the stability and interaction with the biological environment [76]. GNPs of distinct size and shapes can be produced using biological, physical, and chemical means.

In 1951, Turkevich et al. demonstrated a synthetic method for producing GNPs by adding citric acid to hydrogen tetrachloroaurate (HAuCl4) in boiling water [77]. This method was further improved in subsequent studies to control the particle size of GNPs [78]. The biological synthesis of GNPs is a relatively new and promising field. Many plants and microorganisms can participate in the synthesis of GNPs by secreting various enzymes resulting in the reduction of gold ions [79, 80]. Along with effective biocompatibility, harmless, and high surface-to-volume ratio, GNPs have the ability to quench fluorescence [81].

*Quantum dots (QDs)* are nanosemiconductor particles with a core of heavy metal and coating of an organic compound. They are equipped with optical and electronic properties [82]. Major characteristics of QDs are photostability and luminescence. They are used as substitutes to the organic fluorescent dyes in biological sensing and imaging [83]. The top-down processing and bottom-up approaches are used to synthesize QDs. X-ray lithography and ion implantation are the two methods of top-down approaches, and wet-chemical methods and vapour-phase methods are the two methods of bottom-up (self-assembly methods) approaches [84]. Because of high optical characteristics and possible toxicity, QDs are not commonly used for drug release, but instead used as bioimaging agents to observe specific things like ATP and glutathione [85, 86].

*Silver nanoparticles (AgNPs)* are made up of silver atom. Their size ranges from 1 nm to 100 nm. They are extensively used across various fields because of their exceptional chemical and physical characteristics such as optical, thermal, electrical, and biological properties [87]. Their wide range of applications includes antibacterial agents, optical sensors, drug delivery, medical device coatings, anticancer agents, and textiles [88–90]. Their remarkable properties and applications demand various methods for the synthesis of AgNPs. One of the most common methods for producing AgNPs is the reduction of silver salts using reducing agents like Ocimum sanctum [91, 92]. The biologically prepared AgNPs are reported to depict high yield, solubility, and stability. In order to ensure the safety issue, toxicity, or biocompatibility, the various characteristics of nanomaterials must be evaluated [93].

*Carbon* has the atomic number of 6 and has six electrons that fill 1s2, 2s^2^, and 2p^2^ atomic orbitals. It can hybridize to form sp, sp^2^, and sp^3^ orbitals [94]. Carbon nanotubes (CNTs) are tubular sp2 nanocarbon materials made of rolled-up sheets of graphene [95]. CNTs can either be single-walled (SWCNTs) with a diameter of less than 1 nm or multiwalled (MWCNTs) with diameters reaching more than 100 nm [96, 97]. Most of the properties of CNTs are similar to that of graphite. Several techniques have been developed in the synthesis of CNTs such as carbon arc discharge technique, chemical vapour deposition, and the laser ablation technique [94]. While outer walls can be modified with different organic materials, one can make use of the inner hollow core to encapsulate chosen drug for biocompatible targeting purposes [65].

*Silica nanoparticles (SiNPs)* are a distinct group of nanoparticles with a diverse set of properties. Mesoporous silica nanoparticles (MSNs) are the most studied subtype of SiNPs. They contain porous channels of silica particles with an aperture size ranging between 2 nm and 50 nm. MSNs have been largely expended in drug release and biomedical usage [98, 99]. The tunable aperture size and regulated mesoporous structure aid in drug dissolution and further prevent drug crystallization. Because of their biocompatibility, harmless, and biodegradability, SiNPs possess a great potential for medicinal use. The most commonly used producing methods are Stober's process and microemulsion [100]. It is reported that regulated and targeted delivery options can be devised to enhance therapeutic efficacy while reducing adverse and toxic effects [101].

## 5. Nanomaterials in Environmental Remediation

Nanomaterials have higher reactivity and, thus, effectiveness than larger and heavier counterparts owing to its high surface-to-volume ratio. Furthermore, when compared to traditional approaches, nanomaterials have the ability to control distinctive surface chemistry, enabling them to be functionalized or embedded by functional groups capable of targeting particular molecules of concern (pollutants) for effective remediation. The materials that are used in the remediation process must not be another cause of pollution themselves. Therefore, the use of biodegradable materials is exciting in this field of application. Some of the functions of nanomaterials in environmental remediation are shown in Table 2.

### 5.1. Metal-Based Nanomaterials

Metals and metal oxides such as gold, silver, titanium oxide, and iron oxide are the most explored nanoparticles for environmental remediation [114]. AgNPs are recognized for the antibacterial properties and therefore are widely suggested for the treatment of wastewater [102, 103]. Silver ions were reported to alter the cell membrane structure and increase its permeability [105]. Silver ions are shown to improve the UV deactivation of viruses and bacteria because they are photoactive in the incidence of UV irradiation [106]. The size and shape of AgNPs were shown to affect their properties and function. Pal et al. reported that triangular AgNPs displayed better antibacterial results than nanorod AgNPs and nanosphere AgNPs [129]. Current findings have focused on incorporation of AgNPs with other materials like metal oxides and polymers to improve efficiency of the resulting composite [104].

Iron nanoparticles have substituted the use of massive iron-based structures for water treatment. They have been proposed for the groundwater remediation as they were reported to reduce and precipitate metal ions effectively [107]. Gold nanoparticles allow the removal of inorganic mercury present in drinking water. Mercury ions were initially shrunk to zero-valent condition and were then coated on the surface of gold nanoparticles [108, 130].

Metal oxide that is extensively investigated for environmental remediation is titanium dioxide (TiO_2_). TiO_2_ nanoparticles are used in air purification and self-cleaning surfaces along with effluent treatment because of their properties like nontoxicity, semiconductivity, energy conversion, and photocatalytic properties [109, 131]. Rodriguez demonstrated that the composite of gold and TiO_2_ nanoparticles was highly efficient during desulphurization [110]. The nanoparticles are doped with other transition metal ions to increase the photocatalytic degradation. Ag-doped TiO_2_ nanofibers were shown to have increased photodegradation of 2-chlorophenol under UV treatment [111]. In addition, titanates, the inorganic compounds of titanium oxide, were described for the elimination of pollutants [112]. TiO_2_ nanoparticles are also used as a catalyst to convert harmful sulphur dioxide (SO2) from atmosphere into sulphur through a chemical reaction. Therefore, TiO_2_ nanoparticles have been extensively used for the reductive and oxidative conversion of contaminants in the air and the water. Another metal oxide, zinc oxide (ZnO) was used as an adsorbent to remove heavy metals [113]. ZnO showed higher removal rate of copper ions, and ZnO nanosheets were reported to have good capacity of absorbing lead [114]. Furthermore, ZnO is reported to exhibit strong antimicrobial properties towards broad spectrum of bacteria [132]. Different types of nanomaterials involved in environmental remediation are illustrated in Figure 4.

### 5.2. Silica Nanomaterials

Mesoporous silica nanomaterials have several advantages aimed at environmental remediation such as excessive surface area, considerable pore volumes, easy surface modification, and adjustable pore size [115]. Because of their exceptional performance as adsorbents, MSNs have been used in a range of studies for contaminant redress, particularly in the gas segment. Amino-functionalized and thiol-functionalized MSNs have been consumed in the deduction of heavy metals present in wastewater [116]. Amine-modified xerogels of silica nanomaterials were used in treating the pollutants such as carbon dioxide and H_2_S from natural gas [118]. In addition, organic dye removal from wastewater has been reported using silica-based materials. Because carboxylic acid forms hydrogen bonds through various compounds, mesoporous silica was functionalized with various substances like metal ions, pollutants, and dyes for the removal of several metal ions like Al^2+^, Cd^2+^, Co^2+^, and Ni^2+^ [117]. Furthermore, SiO2 nanoparticles have been modified with 2,6 pyrimidine dicarboxylic acid and consumed as a sorbent to deduct mercury ions present in the aqueous solution [119].

### 5.3. Carbon-Based Nanomaterials

Fullerenes, carbon nanotubes, and graphene are the different structural configurations of carbon-based nanomaterials. Various investigations were reported determining their usage for environmental remediation. Brunet et al. demonstrated that tuned hydrophilic fullerenes (C60) can be used to kill toxic microorganisms from water through photocatalytic process [120]. Interestingly, fullerenes were reported to store hydrogen by converting C-C bonds to C-H bonds [120]. The composite from fullerene C60 with polyvinylpyrrolidone is reported to exhibit antibacterial properties and is used in water disinfection. Fullerenes have a possibility to be operated in membrane technology due to their ease of functionalization, high strength, high electron affinity, etc. [121].

CNTs, either SWCNTs or MWCNTs, have been the most studied carbon-based materials for environmental remediation. They can be easily functionalized with other compounds making them a selective and powerful adsorbent [133]. Adsorbent-based purification process is widely applied in the purification of contaminated air and drinking water [134]. Anitha et al. demonstrated that functionalized SWCNTs had higher adsorption capacities towards heavy metal ions like Cu^2+^, Hg2^+^, Cd2^+^, and Pb^2+^ [122]. Furthermore, nanocomposites such as MWCNTs-ZrO_2_, MWCNTs-Fe_2_O_3_, MEWCNTs-AL_2_O_3_, MWCNTs-FE_3_O_4_, and MWCNTs-MnO_2_-Fe_2_O_3_ were effectively used for the deduction of heavy metal ions of As^3+^, Cr^6+^, Pb^2+^, Ni^2+^, and Cu^2+^ [123–126].

Graphene has a thin hexagonal layer of carbon atoms and is said to have immense strength. Tabish et al. fabricated porous graphene that is useful as an adsorbent to remove As^3+^ ions from water with 80% efficiency [127]. The reduced graphene oxide was functionalized for the deduction of different heavy metal contaminants present in the aqueous solution like Pb^2+^, Cu^2+^, Cr^3+^, and Cd^2+^ [128]. Likewise, several studies were conducted to design nanocomposite of graphene with various compounds and employed them for the deduction of different heavy metal ions present in water.

## 6. Limitations of Nanomaterials in Environmental Remediation

Although nanomaterials have remarkable properties such as high efficiency and reactivity, they have limitations that prevent them from being used on a large scale in environmental remediation. It is believed that they have adverse effects on the environment. Their toxicity and following effects on the ecosystem and human health are the leading concerns. Along with the aforesaid risks, challenges in the regeneration and reuse of nanomaterials will greatly affect the cost of the treatment. Furthermore, the harsh and toxic conditions in environmental applications would degrade the structure of the nanosized particles used. Besides that, there is a need for a well-defined classification of nanomaterials used in environmental remediation for a better understanding of the diverse properties and functions of nanomaterials.

## 7. Future Directions

In addition to the efforts concerning the well-being of the patients and dentists at the dental clinics [135, 136], several attempts have been made in investigating different techniques for providing better oral care. One such advancement is the incorporation of nanomaterials into dentistry. Future advancements in addressing unsolved problems related to dental materials would involve using antimicrobial concepts utilizing nanomaterials or nanocoatings, improved nanoceramics, development of hybrid dental implants, and nanobiosensing systems, which would enhance their structural reliability and damage control. Moreover, nanobiomineralization methods are said to have a significant impact on the regeneration of dental hard tissues, and this topic is expected to grow in the future.

Nanomaterials provide many advantages, such as greater sensitivity, real-time detection, smaller sample sizes, portability, and lower cost in environmental remediation. In addition to metals and metal oxide nanomaterials, nanomembranes have found applications in water treatment. Nanofibers and nanocomposites have recently been proposed as effective in the adsorption of pollution from wastewater. However, the large-scale production and more widespread application of these nanomaterials still remain unexplored. There is a room for improvement in the production of nanomaterials that can selectively remove pollutants, have greater resistance and stability, and are less toxic.

## 8. Conclusion

It is evident that nanoparticles greatly influence dental research and treatment procedures, leading to better oral health care in the near future. There is a plenty of room for the development and improvement of dental materials using nanotechnology and its new fields of applications in dentistry. Consequently, there is a pressing concern about the release of heavy metal wastes from dental clinics. Nanoparticles may provide a more sustainable and comprehensive approach to addressing this serious issue. However, there is still need for further improvements regarding nanotechnology for environmental remediation. Most of the studies were carried out in the laboratory settings, and thus, multitudinous studies are required in real case scenario to fully understand how nanomaterials can significantly help in environmental remediation.

## Figures and Tables

**Figure 1:** Key sources of pollution caused by heavy metals in dentistry. Created using BioRender.

**Figure 2:** Various fields of dentistry currently using nanoparticles. Created using BioRender.

**Figure 3:** Classification of nanomaterials. Created using BioRender.

**Figure 4:** Different types of nanomaterials involved in environmental remediation. Created using BioRender.

**Table 1:** Current functions of nanoparticles across various branches of dentistry.

Dental branch	Nanomaterials	Applications	References
Periodontics	Triclosan-loaded nanoparticles	Treating periodontal inflammation	[29]
	Nanoparticle-delivered enzymes	Remodelling periodontal fibres	[30]
	Nanostructured doxycycline gel	Repairing periodontal surface	[31]
	Nanorobots	Antibacterial properties	[32]

Endodontics	Chitosan/zinc oxide/silver-based nanoparticles	Disinfection of microbes	[33]
	Nanoassemblies of polyglutamic acid and poly-l-lysine	Reduce dental pulp inflammation and promote regeneration of pulp fibroblasts	[34,35]

Orthodontics	Silver/titanium oxide-based nanoparticles	Antibacterial properties	[36]
	Fullerene-like nanoparticles	Act as dry lubricants to reduce the friction on orthodontic wires	[37]
	Alumina-based nanomaterials	Increase strength of plastic polymer braces	[38]

Prosthodontics	Zirconium dioxide/alumina-based nanoparticles	Increase flexural strength	[39]
	Titanium dioxide-based nanomaterials	Reduce porosity of denture material	[40]

Restorative dentistry	Hydroxyapatite	Used as fillers to repair small dents on enamel	[41]
	Calcium phosphate	Used as filler on enamel	[42]
	Bioactive glass	Dentin mineralization	[43]
	Chitosan-based nanoparticles	Drug delivery and improved affinity towards enamel	[44,45]
	Nanofibers-based scaffolds	Dental pulp regeneration	[46]

**Table 2:** Nanoparticles and their applications in environmental remediation.

Nanomaterial	Application	References
AgNPs	Treatment of wastewater due to their antibacterial properties	[102–104]
Ag2^+^	Affect cell structure and permeability of cell wall	[105]
AgNPs	Act as photocatalyst and increases the UV inactivation of bacteria and viruses.	[106]
Iron nanoparticles	Groundwater remediation by reducing metal ions effectively	[107]
Gold nanoparticles (AuNPs)	Remove inorganic mercury from drinking water	[108]
Titanium dioxide (TiO_2_)	Air and wastewater purification	[109]
Gold and TiO_2_ composite	Efficiently removes sulphur	[110]
Silver-doped TiO_2_ nanofibers	Photodegradation of chlorophenol	[111]
TiO_2_-based nanoparticles	Removal of harmful sulphur dioxide from air	[112]
Zinc oxide	Adsorbent to remove heavy metals such as copper and lead	[113, 114]
Mesoporous silica nanomaterials (MSN)	Excellent adsorbent to remove pollutants from the air	[115]
Amino/Thiol-functionalized MSNs	Removal of heavy metals from wastewater	[116, 117]
Amine-modified xerogels	Removal of carbon dioxide and H_2_S from natural gas	[118]
SiO_2_	Removal of mercury from aqueous solution	[119]
Fullerenes (C60)	Used to kill microbes via photocatalytic process	[120]
Composite of fullerene and polyvinylpyrrolidone	Used in water disinfection by killing bacteria	[121]
SWCNTs	Adsorption of heavy metals	[122]
MWCNTs	Removal of heavy metal ions	[123–126]
Graphene	Adsorption of heavy metal contaminants from wastewater	[127, 128]

## Data Availability

The data used to support the findings of this study have not been made available because no new data were generated.
